# A Fine-Tuned BERT-Based Transfer Learning Approach for Text Classification

**DOI:** 10.1155/2022/3498123

**Published:** 2022-01-07

**Authors:** Rukhma Qasim, Waqas Haider Bangyal, Mohammed A. Alqarni, Abdulwahab Ali Almazroi

**Affiliations:** ^1^Dept. of Computer Science, University of Gujrat, Pakistan; ^2^University of Jeddah, College of Computer Science and Engineering, Department of Software Engineering, Jeddah, Saudi Arabia; ^3^University of Jeddah, College of Computing and Information Technology at Khulais, Department of Information Technology, Jeddah, Saudi Arabia

## Abstract

Text Classification problem has been thoroughly studied in information retrieval problems and data mining tasks. It is beneficial in multiple tasks including medical diagnose health and care department, targeted marketing, entertainment industry, and group filtering processes. A recent innovation in both data mining and natural language processing gained the attention of researchers from all over the world to develop automated systems for text classification. NLP allows categorizing documents containing different texts. A huge amount of data is generated on social media sites through social media users. Three datasets have been used for experimental purposes including the COVID-19 fake news dataset, COVID-19 English tweet dataset, and extremist-non-extremist dataset which contain news blogs, posts, and tweets related to coronavirus and hate speech. Transfer learning approaches do not experiment on COVID-19 fake news and extremist-non-extremist datasets. Therefore, the proposed work applied transfer learning classification models on both these datasets to check the performance of transfer learning models. Models are trained and evaluated on the accuracy, precision, recall, and F1-score. Heat maps are also generated for every model. In the end, future directions are proposed.

## 1. Introduction

Natural language processing is a scientific process to train a computer to understand and process human language. NLP gained a lot of importance in recent years because of the researchers and processing powers of machines. Researchers are doing their best to generate interesting facts and figures from human language and implement those results in every field of life from educations to hospitals, industry to shopping malls, etc. In past, NLP problems were solved using rule-based systems. However, due to the different nature of text in the world, machine learning is applied to NLP and it has gained a strong ground using SVM and Naïve Bayes. Natural language processing and text mining refer to the process of human-generated text that came from multiple social media networks using different algorithms, programs, and techniques. It is an important field of AI. With continued research on text mining and NLP using data mining algorithms, machine learning, and deep learning, data mining techniques have gained the best results in the fields of automatic question answering machines, anaphora resolution, automatic abstraction, bioinformatics, and web relation network analysis [1]. Researches show that NLP, data mining, and text classification can be very helpful in every prospect of life. There are also many other researchers who have used NLP in hate speech, sentiment analysis [2], detection of controversial Urdu speeches [3], movie reviews [4], stock market [5], online reviews [6], and restaurant reviews [7].

In recent decades, social media has gained huge importance because of its usage for different purposes. If people use social media often, then it is obvious they will generate a huge amount of data. Because of this huge data generated by social media users, hate speech is also increased. For example, if a movie is released, the audience will have good or bad or neutral reviews or comments about it. Researchers had also done plenty of work in the area of hate speech as well and it is increasing day by day. The paper [8] had explained how NLP is involved in hate speech tasks and how it is able to automate the process to capture and detect hatred social media content. These researches involve NLP as they are using human-generated natural content. Social media content generated by social media platform users is an important source of data for hospitals, industry, scientists, policy-making, and much more. UGC (User Generated Content) on different review platforms or sites holds diverse information in the form of text that is extracted after applying opinion extraction algorithms and sentiment analysis techniques [9] These algorithms provide better performance in the feature extraction phase of text classification as well [10–24].

A group of researchers had worked and highlighted the limitations and gaps in the field of hate speech [25]. A solution to reduce these limitations was also proposed. They had elaborated that a large amount of sufficient data to train an automated approach. Insufficient labeled data related to hate speech is a big problem in the detection of hate speeches on social media. Their proposed approach was pretrained on BERT. One of the important tasks in hate speech detection is to categorize portions of text based on their context and make developers capable of text classification tasks in NLP [26]. Their trained model on the Italian hate speech dataset is named as ALBERTo. This model is highly sensitive regarding the temporal distances of datasets. But its main advantage is as follows: after a time, its performance increases, and it required less training data than previous classifiers. Hate speech and offensive languages are two different things. Separating hate speech from offensive language is a difficult task [27]. Their research uses a crowdsourced lexicon of hate speech to collect tweets and then label them as offensive, hateful, and neutral metaheuristic algorithms which are used for text and data classification tasks [80, 82, 90].

Transfer learning is a phenomenon or task in which the information gained from unlabeled data can be used in relative tasks with a small labeled dataset. And that small labeled dataset achieves high accuracy with the help of previous information. NLP transformers have gained promising accuracy in every practice as compared to ML and DL techniques. They have written in their research that the key idea behind TL is to grab information from related areas to help systems based on machine learning to obtain higher accuracy in the area of interest. Thus, we can also say that transfer learning can also be used to achieve high performance with less human supervision as compared to active learning and supervised learning. There are many examples in our real life which we can relate to transfer learning. For example, if a system is already trained to recognize apples, then it may be also used with little fine-tuning to recognize pear as well. This will need less data and less training time. The key idea behind transformers is attention.

Social media has a great empowerment impact. Every user can post based on their thoughts. They trained already existing models to predict the posts or news related to coronavirus as real or fake. Among all trained models, transformers showed the best results. News is a great source and holds great importance as they keep everybody updated. Fake news took birth in the 18^th^ century [28]. The Internet makes it easier to spread fake news through the excessive use of social media. It is also very tough to distinguish between real and fake news. Already existing approaches have deficiencies which they tried to overcome by developing a hybrid approach.

The rest of the paper is organized as follows.  Section 2 discusses the literature review.  Section 3 discusses the types of classification algorithms.  Section 4 overviews methodology. Experimental results are discussed in Section 5. The conclusion and future prospects of our work are discussed in Section 6.

## 2. Literature Review

Transfer learning nowadays holds spectacular importance in the research area. Researchers are trying hard to achieve higher accuracies in every research by applying different versions of transformers. A team of researchers [29] performed a comprehensive survey of sentiment analysis in finance in which they have evaluated recent researches and advancements regarding finance. They have evaluated techniques including lexicon-based approaches for text classification, statistical methods, sentence encoders, word encoders, and transformers. Their evaluation of the finance dataset clearly shows that transformers outperformed among all existing methods and techniques with the highest accuracy. They have applied different models of transformers including BERT, FinBERT, XLNet, XLM, ALBERT, RoBERTa, DistlBERT, XLM-RoBERTa, and BART. All these transformers gained a high *F*1 score among all. Between these NLP transformers, BART launched by Facebook achieved the highest *f*1 score of 0.85.

Researchers performed an evaluation of sentiment analysis approaches based on transfer learning for the Japanese dataset [30]. They have performed binary sentiment classification and multisentiment classification on product reviews and movie reviews. After their research, they have stated that transfer learning approaches perform way better than models that are generated for task-specific purposes on 3 times greater data. They have stated that better systems exist for the English language but there is much deficiency for the Japanese data. So, they tried 3 transfer learning models including BERT, ELMo, and ULMFit. All these models have achieved less error percentages compared to other models using datasets including the Rakuten dataset and Yahoo movie review dataset. BERT-base gained the lowest rate of 8.42 on the Yahoo movie review dataset and 4.68 on the Rakuten dataset.

These researchers performed a study on the most recent advancements of transfer learning in the field of natural language processing [31]. Firstly, they have checked recent machine learning and deep learning approaches and then also checked recent TL approaches. They have noticed that transfer learning approaches have brought new dimensions for different NLP tasks. Transfer learning can be happily and effectively used in the areas where we have less data to train. We can use a pretrain model and then fine-tune it. They have experienced that transfer learning models can perform better than other state-of-the-art methods in NLP. BERT is trained on BookCorpus, text corpus, and Wikipedia which can give overwhelming results in some areas of natural language processing but it still needs to be improved [32]. It somewhere lacks domain-related and task-related knowledge. It is where improvement is required. They have presented a new version of BERT called BERT4TC BERT for text classification. Their model is rich in sense of domain- and task-related knowledge. They have evaluated their proposed model on publicly available datasets. Results showed that the model they have proposed with compatible auxiliary sentences outperforms compared to both feature-based typical methods and some fine-tuned methods and achieved new state-of-the-art results in multiclass classification.

This research proposes a political sentence-level text classifier using human experts' annotated corpus for political manifestos [33] and then applied to press briefings of COVID-19. They have manually annotated the manifestos as training data on a classifier and then applied that to press briefings to automatically classify existing sentences in press briefings. They have combined CNN with BERT transformer, and it showed that CNN combined with BERT gained the highest accuracy among other models compared with CNN. They have done four experiments named M1, M2, M3, and M4. M4 performed better among all as it is CNN + BERT. It contained high accuracy and an *F*1 score. Fine-tuning of desired pretrained models is an efficient transfer mechanism. However, fine-tuning may be inefficient in some tasks and need to build entire new techniques for solving multinature problems [34]. As an alternative to it, they have proposed an adapter module with the transfer. These modules generate an extensible model. We only need to add a few parameters which are trainable on every task, and we can add a new task without revision of the previous one. Parameters that are from the original model remain fixed with high parameter sharing. They have evaluated BERT on 26 different classification tasks. And they have used GLUE as a benchmark. GLUE achieved high performance with full fine-tuning of parameters by adding only 3.6% parameters per task. Fine-tuning trains 100% of the parameters.

Evaluation of deep learning approaches and transfer learning approaches for fake news detection using COVID-19 fake news detection dataset (consisting of 10,700 social posts and articles) was performed by [35]. They used classification algorithms bi-LSTM + Attention, HAN (hierarchal attention network) BERT-base, and DistilBERT. Their aim is to classify the news as fake or real. The fake news detection task is formulated as a text classification problem. They rely on the content of the news and ignore other important features like user characteristics, social circle, etc. which might not always be available. The BERT and DistilBERT models pretrained on the COVID-19 tweets corpus perform better than the ones which are only fine-tuned on the dataset. The BERT-cased model which was trained manually on the COVID-19 tweets corpus gives the best results followed by the COVID-Twitter-BERT model. Reference [36] elaborated the impact of social media in our daily lives. They also highlighted the misleading information on social media and its effect on our lives. They proposed an approach to detect the fake and real news about COVID-19. The model achieves high *F*1 score and occupied the second position on the leaderboard. They used the dataset containing posts and tweets collected from Facebook, Twitter, and Instagram. They have split the dataset into train test and validation parts. They tried different baseline models on this dataset and also used different transformer models. And results clearly show that their RoBERTa model achieves a 0.9864 *F*1-score and their Electra model achieves a 0.9827 *F*1-score on the official test set.

This research highlights the impact of fake news related to coronavirus [37]. They stated that most social media posts are not trustworthy as they lead the readers toward wrong information that can cause panic situations among people. They presented their results on COVID-19 Fake News Detection in English and achieved the first position in the leaderboard among 166 submitted results. Their proposed model uses CT-BERT (COVID-Twitter-BERT) and achieves a 98.69 *F*1-score. Their research developed a method to check the reliability of social media posts that belong to COVID-19 [38]. They ensemble three transfer learning models (BERT, ALBERT, and XLNET) for classifying COVID-19 news into real and fake. They have used the COVID-19 Fake News Detection in English dataset. Their proposed methodology achieves a 0.9855 *F*1-score on the test set and among 160 teams getting the 5^th^ rank. They split the dataset into training, validation, and testing parts for the experimental setup.

A multimodal approach for fake news detection was developed by [39]. Because in past years, posting wrong, hateful, abusive, offensive, and hateful content on social media tools has increased in exponential format, people spread their inner negativity related to any situation on social media. This may lead other people toward a wrong and hateful path. That is why it is the need of the hour to detect those profiles and people who do this sinful act. Researchers used different strategies to accomplish this purpose. The authors of this research work propose a multimodal approach based on multi-image. In specific, their system uses textual, semantic, and visual data or information. They had used BERT for textual data to extract the semantic and contextual meaning of the text. They further used the VGG-16 model for visual representation and tag extraction. And the rest of the semantic information is calculated using cosine similarity. They had used GossipCop, a part of the FakeNewNet dataset. This multimodal multi-image approach achieved a 0.7955 *F*1 score on testing. This approach had also increased the performance of baseline models.

With the rapid growth of social media in past years, it has become more convenient for people to access news fast than ever. They said that it is also happening that people are spreading fake news over social platforms for their own purposes. Many researches using supervised learning had been proposed to detect fake news. These approaches focus on different features to make the classification more accurate like news content, social context, user profile, and messages context. These approaches showed accuracy but face limitations as they need a reliable accurate dataset [40]. Their proposed work was an unsupervised framework called the Unsupervised Fake News Detection Technique (UFD) to minimize this problem. They mainly focused on two aspects: user's reliability and truth of news to filter the fake news among real news. They had tested their framework on datasets which are LIAR containing 12,800 short news statements, and BuzzFeed has 1,627 news articles related to U.S. elections. But they used 332 and 144 after filtering datasets. UFD achieved the highest accuracy, precision, recall, and *F*1-score on both datasets. The model achieved 0.759 and 0.679 of accuracy on LIAR and BuzzFeed, respectively.

Nowadays, society is more and more connected and attracted to the Internet. People around the globe make it a necessary part of their lives. Information we retrieve and gather from Internet has become an essential part of our lives [41]. They had described that this extra dependence on Internet has led us to its wrong impacts as well, as it is leading us toward hatred, abusive, offensive, and toxic language. Machine learning is doing great in the field of NLP. They had developed the DeepHate model for text analysis which is trained on several small datasets to make it more accurate. Their model can learn a single hate speech pattern from unrelated and diverse data sources. The model works on transfer learning and can generate both word representation and sentence representation. They used an English tweets dataset containing 37,520 tweets. Another dataset is also used containing 22,304 tweets including offensive, hateful and harmless tweets.

## 3. Types of Classification Algorithm

This research work uses machine learning and transfer learning classification algorithms. These models are applicable to many natural processing tasks and work efficiently on these tasks. The following mentioned models are used in this research procedure.

### 3.1. BERT-Base

Bidirectional Encoder Representation from Transformers (BERT) was proposed by [42]. The main purpose of BERT is to train bidirectional representations from an unlabeled dataset. It works on collaborative left and right context phenomena in all layers. BERT is simple yet powerful. It generates promising results in several machine learning tasks. A fine-tune model of BERT only needs to add one more layer for each new model to perform a variety of tasks. It uses a masked language model. MLM works on the phenomena of masking random words from input and then it predicts the ID of that word by utilizing its context. MLM uses both left and right contexts which enables training of the bidirectional model. They joint MLM with next sentence prediction (NSP) as well. BERT-base is comparatively smaller in its size, it takes less time for computation and processing, and also it is affordable. It is not applicable to ambiguous data mining or text mining tasks. Reference [43] used it in the detection of fake news. The paper [44] used it for content enhancement and it proves its promising results in content enhancement field. It was also used by [45] for distilling its knowledge. Reference [46] performed sentiment analysis using BERT and it has done a great job there as well.

### 3.2. BERT-Large

BERT-large is a type of BERT model. It works similarly as BERT-base does but it has a larger size than BERT-base. It is more expensive than BERT-base as it takes more time for computation and is applicable to large datasets. The article [47] used BERT-large in his research work to process the COVID-19 related content on Twitter. BERT-large performed well on his dataset but his proposed approach performed better. The paper [48] used BERT-large in offensive tweet classification, and among all evaluated approaches, BERT-large stands the second on a scale with a 0.781 *F*1 score. The authors of [49] performed multiple experiments on deep learning and transfer learning approaches to access syntactic abilities and they have seen that between all approaches BERT-based transformers performed extremely well.

### 3.3. RoBERTa-Base

The authors of [50] proposed RoBERTa model with slight advancements in BERT which are as follows: training their model with more data and larger batch size, eliminating the next sentence prediction factor, having larger sequences, and making changes in masking pattern. Their proposed model performs well in many experimental setups. They have also noticed that the linguistic bias of RoBERTa-base is stronger. Roberta uses BookCorpus, OpenWebText, English Wikipedia, STORIES, and CC-News. The authors of [51] did research on learning features that are also important. They explained that RoBERTa obtains linguistic generalization as preferences. Reference [52] compared three methods including LSTM, BERT, and RoBERTa for detecting and classifying mental illness on multiple social media platforms. And RoBERTa outperforms among these three approaches. Reference [53] used RoBERTa to classify informative tweets related to COVID-19 and their approach showed the best results.

### 3.4. RoBERTa-Large

Reference [54] applied RoBERTa-large with dialog history attention to select the responses based on a randomly wired network. Research has shown that the RoBERTa-large model needs more computer resources than RoBERTa-base. That is why it is not widely used by researchers. The article [55] used RoBERTa to highlight and detect medications on Twitter. They used an unbalanced dataset and their proposed model achieved a 0.8 *F*1 score. The paper [56] used RoBERTa for a Dutch language model. Their experimentation showed that training a BERT model on the Dutch language shows a lot of variety in multiple tasks for the Dutch language. The authors of [57] used RoBERTa-large for eye-tracking prediction. And their technique showed promising results with a 3.929 MAE score and stands in 3^rd^ position among 13 teams.

### 3.5. DistilBERT

DistilBERT was introduced in 2019 by [58]. It was a lighter, fast, smaller, and cheap version of BERT with a size reduction of 40% with 60% more speed and 97% understanding of language capabilities. This lighter and useful version was used by many researchers. The authors of [59] used this lighter version of BERT for sociopolitical news classification. DistilBERT showed promising results in their experiments. The authors of [60] combined linguistic knowledge with different transfer learning models to enhance their performance. And their methodology worked really well in this perspective. Ensemble models boosted the performance of used models by many points. The authors of [61] used this version of BERT for detecting health information along with named entity recognition tasks. And the detection was improved by half which was promising. The authors of [62] worked with DistilBERT and proposed a mechanism for answer selection and picking up important words. The performance was improved by 0.6% which is not bad at all. The authors of [63] retrained DistilBERT on universal dependencies for the purpose of a voice shopping assistant. The performance of these downstream tasks is raised by 1.31%.

### 3.6. ALBERT-Base-v2

With the collaboration of Toyota Technologies and Google Research, they jointly released the scalable and smaller successor of BERT in 2019 which they named ALBERT [64]. It mainly involved reduction in two parameters: increase in training speed of BERT and lower memory consumption. ALBERT performs better in multiple classification tasks. It also uses a very low number of parameters while doing sentiment analysis. The authors of [65] used the ALBERT transformer approach for contextualized sarcasm-based detection on Twitter. They have applied other transformer approaches as well. The authors of [66] also evaluated this model for fake news detection and additionally checked the facts for these fake news which worked really well and lead among all models. The authors of [67] checked this approach for question answers on COVID-19. ALBERT gained the highest exact match score of 13.04. The authors of [68] used ALBERT for medication prescriptions used on social media.

### 3.7. XLM- RoBERTa-Base

The authors of [50] proposed this model and trained it on hundred languages with two TB of data which was filtered. Their model which was combined with XLM-R outperforms with 23% accuracy compared to many transformers. The authors of [69] identified offensive language using this ensemble technique. They joint XLM-RoBERTa with DPCNN, and this model showed amazing results. These two also used this approach for hope speech detection attention, and this shows promising results in this task. They achieved 0.59, 0.84, and 0.92 *F*1 scores for Tamil, Malayalam, and English languages. The authors of [70] used this and experiment with it for multilanguage sentiment analysis. And the model achieved a good *F*1 score. The authors of [71] performed another research work of classification using neurons for the task at EVALITA 2020. They had used the hate speech dataset and performed the experiment. The model achieved a 0.798 *F*1 score. The authors of [72] used XLM-RoBERTa for context disambiguation in words. The model outperforms all experimented methodologies.

### 3.8. Electra-Small

BERT uses Masked Language Modeling and replaces some tokens with masks and then reconstructs the model using these masks. But this requires a large amount to compute, so the authors of [73] proposed Electra and overcome this issue. Their proposed approach replaces tokens with alternative samples. And after that, they did not train the model; they made sure that each token in input is swapped with a sample generator or not. The authors of [74] used Electra for profiling fake news. They have created an ensemble model considering 15 models. Then, they are fined tuned according to the tasks and dataset. Electra achieved 0.70 and 0.69 *F*1 scores for English and Spanish datasets, respectively. Electra was also trained with multiword selection by [75].

### 3.9. BART-Large

Facebook researchers in October 2019 proposed BART [76]. The formation of BART is similar to BERT and GPT2. Tasks like question-answer and summarization of any text are done accurately. This model showed promising results in these kinds of tasks. This one takes advantage that the encoder and decoder form BERT and GPT AR, respectively. It considers the autoregressive techniques to check dependencies which makes it better than BERT. Its encoders and decoders are connected. They used BART for an automated speech recognition system. They had done the experimentation for 1000 hours on the speech recognition dataset and they have reduced the error rate to 21.7% which is a huge success and way better than the baseline model. The authors of [77] used it for supervised topic label generation. Their model performs better than the baseline model. The authors of [78] also evaluated this model for query suggestions. Their proposed approach has a better understanding of noise and can handle and understand complex queries. The authors of [79] performed visual common sense generation and called it Knowledge Enhanced Multimodal BART. The authors of [80] evaluated BART for knowledge grounded conversation tasks and achieved good results.

## 4. Methodology

Due to the complex nature of social media data on COVID-19 fake news and hate speech, it is quite obvious that the proposed model must have different aspects to precisely and accurately predict the fake and real news and similarly hateful or nonhateful content.  Figure 1 elaborates the steps and architecture of the fine-tuned model.

### 4.1. Data Sets

Two datasets are used in this research work. The first is named “COVID-19 fake news dataset” which was originally generated in 2020 by Sumit Bank and was published and made freely available on Coronavirus Disease Research Community-COVID-19. It contains 10202 fake news related to coronavirus which different users shared on social media sites. Some of them are gathered from Facebook, some belong to Instagram, and others belong to websites and Twitter blogs. All of them are collected using different keywords including COVID-19, pandemic, corona, and coronavirus. This dataset is basically assembled in two columns. The first contains text, special characters, and attributes which is named as Title, and the second contains binary values as 0 and 1 and named Outcome. Here, 1 presents real news while 0 presents fake news.

The second dataset which is used in this research work is named “extremist-non-extremist dataset” which was developed by [81]. The dataset was generated using Twitter streaming API, and tweets containing more than one extremist word like ISIS, suicide, bomb, etc. are collected. Each review is compared with seed words present in a manually built extremist lexicon and added to the dataset. The final data was stored in a .csv file. The dataset consists of 21,186 tweets in total, of which 12,755 are labeled as extremist and 8,432 are labeled as nonextremist. Extremist tweets are replaced with 1 and nonextremist tweets are replaced with 0.

The third dataset which is used in this research work is named “COVID-19 English tweets” developed by [82]. A research had revealed that data which is shared on social media sites is uninformative. Therefore, they thought that informative data should be highlighted through a shared automated task, where all the participants have to use their developed dataset of COVID-19 English tweets. They collected tweets using Twitter API with ten keywords including “coronavirus”, “covid-19,” “covid_19,” “covid-2019,” “covid19,” “covid2019,” “covid_2019,” “coronaVirusUpdate,” “coronavid19,” and “SARS-CoV-2.” Every tweet in the corpus contains a minimum of one word from the above-mentioned keywords. They collected tweets of four months from March 2020 to June 2020. Then, they applied different filters to tweets like removing tweets containing 9 words and also removing the tweet of a person who has less than 5 followers and removing tweets that are retweeted. They have also labeled them as Informative and Uninformative. Informative tweets must contain suspects, death, affected cases, recovered cases, and a number of tests, etc. Train file contains 4820 tweets, test file contains 1539 tweets, and validation file contains 566 tweets.

### 4.2. Data Preprocessing

COVID-19 fake news, COVID-19 English tweets, and extremist-non-extremist datasets which are used in the proposed research work need to be cleaned in the very first step of natural language processing which is called preprocessing step. In this step, cleaning methods on both datasets are applied to remove URLs, converting every word to lower case, and lemmatization and punctuation removal are performed. These methods will eliminate special characters, hyperlinks, empty spaces, identifiers, and words that are very short. This step will clean both datasets.

### 4.3. Encoding

Many efficient and automatic learning models do not accept input in text form. Therefore, the text is converted into digital vectors which rely on the technique of bag-of-words for transfer learning models. We have counted every word's score, and then, feature extraction was also performed. This research work uses the best, efficient, and appropriate classification algorithms based on results from literature reviews and then builds our model accordingly.

### 4.4. Model Evaluation and Testing

After the training model was evaluated and its performance is measured using different parameters including confusion matrix, accuracy, recall, precision, and *F*1-score, we have tested our model on both datasets which are unclassified on fake news, COVID-19 tweets, and hate speech.

Performance evaluation is performed using four parameters which are precision, recall, *F*1-score, and accuracy. Confusion matrix and heat maps are also generated for evaluation purposes. Precision is known as positive values which are gained from prediction. So, it is the fraction of relevant occurrences among gained occurrences. On the other hand, recall is called sensitivity; it is the relevance of gained occurrences. The weighted average of precision and recall is defined as *F*1-score. It takes false positives and false negatives into account. The total number of rightly predicted values is called accuracy. Performance of any classification model is measured using the *N* × *N* matrix which is known as the confusion matrix. It contains true positive, true negative, false positive, and false negative values in the matrix which is used to evaluate the actual values with the values predicted by the classifier. Heat maps are used to observe the data through visualization. It presents different attributes. Visualization helps to find patterns and also gives a perspective of depth. So, heat map is used to explore and observe the data.

This research work uses nine classification models. These classifiers are BERT-base, BERT-large, RoBERTa-base, RoBERTa-large, DistilBERT, ALBERT-base-v2, XLM-RoBERTa-base, Electra-small, and BART-large.

Tables 1–3 present sample tweets for all three datasets. Tables 4–8 show results of nine transfer learning models which are validated using the above-mentioned performance metrics named precision, recall, *F*1-score, and accuracy on COVID-19 fake news dataset, COVID-19 English tweet dataset, and extremist-non-extremist dataset, respectively. Results clearly show that transfer learning classification models outshine using test datasets obtained from reliable sources. Tables 5, 7, and 9 present a comparative analysis for all three datasets with state-of-the-art approaches.  Figure 1 presents the research methodology for the proposed research work. Figures 2–4 show accuracies graph of TL classifiers for COVID-19 fake news, COVID-19 English tweet, and extremist-non-extremist dataset Figures 5–13 present the heat maps for COVID-19 fake news dataset. While Figures 14–22 present the heat maps for transfer learning classifiers and Figures 23–31 show heat maps for extremist-non-extremist dataset.

## 5. Experimental Results

### 5.1. Results for COVID-19 Fake News Data

#### 5.1.1. Discussion

The above-mentioned diagrams and tables contain results for transfer learning classifiers for the COVID-19 fake news dataset. These nine transfer learning classifiers showed excellent performance on the COVID-19 fake news dataset. These classifiers are evaluated using different values of precision, recall, accuracy, and *F*1-score. Transfer learning classification models performed really well and achieved the highest accuracies. Among all transfer learning models, the RoBERTa-base model achieved the highest accuracy of 99.71%. The RoBERTa-large gained the second position and BERT-base achieved the third position among all transfer learning models with 99.68% and 99.56% of accuracy. DistilBERT, BERT-large, BART-large, XLM-RoBERTa, Electra-small, and ALBERT-base-v2 achieved 99.41%, 99.31%, 99.31%, 99.22%, 99.17%, and 98.68% of accuracies, respectively. So, RoBERTa-base leads all seventeen classification models.

#### 5.1.2. Comparative Analysis with State-of-the-Art Approaches

In Table 5, the proposed work is compared with state-of-the-art approaches [83–86] w.r.t to the text classification task. State-of-the-art approaches use machine learning and deep learning techniques including XGBoost, Naïve Bayes, deep neural network, and T1-convolutional neural network. The objective and purpose of experimentation are to perform fake news text classification using state-of-the-art techniques and transfer learning-based proposed fine-tuned approaches. The performance of experimented approaches is compared in terms of accuracy on COVID-19 fake news dataset. XGBoost exhibits the lowest accuracy of 75% on the COVID-19 fake news dataset. The proposed approach achieved the highest accuracy of 99.66% using RoBERTa-base.

### 5.2. Results for COVID-19 English Tweets Dataset

#### 5.2.1. Discussion

Transfer learning models work outstandingly on all experimented datasets and surprisingly take less time.TL models performed best on the COVID-19 tweet dataset. Bart-large won this time with a 98.83% accuracy score. It also performed well in terms of precision, recall, and F1-score as it has achieved 98.85, 98.80, and 98.82 respectively. XLM-RoBERTa stands in the second position with a 98.57% accuracy score. BERT-base and BERT-large gained the third position with a 98.44% accuracy score. They have achieved 98.42 precision, 98.45 recall, and 98.43 F1-score. DistilBERT, ALBERT-base-v2, RoBERTa-large, RoBERTa-base, and Electra-small achieved 98.31, 97.78, 97.00, 96.48, and 94.52 accuracy score, respectively. So, transfer learning models performed outstandingly on all three experimented datasets.

#### 5.2.2. Comparative Analysis with State-of-the-Art Approaches

In Table 7, the proposed work is compared with state-of-the-art approaches [87, 88] with respect to the text classification task. State-of-the-art approaches use machine learning techniques including multilayer perceptron and support vector machine. The objective and purpose of experimentation are to perform tweets classification using state-of-the-art techniques and transfer learning-based proposed fine-tuned approaches. The performance of experimented approaches is compared in terms of accuracy on the COVID-19 English tweet dataset. MLP exhibits the lowest accuracy of 0.78% on the COVID-19 English tweet dataset. The proposed approach achieved the highest accuracy of 98.83% using BART-large.

### 5.3. Results for Extremist-Non-Extremist Dataset

#### 5.3.1. Discussion

All these figures and tables clearly show the performance of transfer learning classifiers on the extremist-non-extremist dataset. Evaluation metrics consist of precision, recall, *F*1-score, and accuracy. Transfer learning classifiers overshine with the highest accuracies. BERT-base and BERT-large shine among other transfer learning models. Both classifiers gained a 99.71% accuracy score. RoBERTa-based gained a 99.6% accuracy score, XLM-RoBERTa and BART-large gained a 99.56% accuracy score, DistilBERT gained a 99.51% accuracy score, RoBERTa-large gained a 99.36% accuracy score, ALBERT-base-v2 achieved a 98.97% accuracy score, and Electra-small gained a 98.73% accuracy score. From all the above-mentioned results, BERT-base and BERT-large both outshine among all nine text classification models.

#### 5.3.2. Comparative Analysis with State-of-the-Art Approaches

In Table 9, the proposed work is compared with state-of-the-art approaches [89–92] with respect to the text classification task. State-of-the-art approaches use machine learning and deep learning-based techniques including Naïve Bayes, CNN, and HDLTex. The objective and purpose of experimentation are to perform tweets classification using state-of-the-art techniques and transfer learning-based proposed fine-tuned approaches. The performance of experimented approaches is compared in terms of accuracy on the extremist-non-extremist dataset. HDLTex achieved the lowest accuracy of 76.5% on the extremist-non-extremist dataset. The proposed approach achieved the highest accuracy of 99.71% using BERT-large and BERT-base.

## 6. Conclusion

In this research, nine transfer learning models which are BERT-base, BERT-large, RoBERTa-base, RoBERTa-large, DistilBERT, XLM-RoBERTa-base, ALBERT-base-v2, Electra-small, and BART-large are applied on COVID-19 fake news dataset, COVID-19 English tweet dataset, and extremist-non-extremist dataset for binary text classification. The experimentation is performed on these datasets which are taken from reliable repositories. All transfer learning models are evaluated using evaluation metrics: accuracy, precision, recall, and *F*1-score.

In the future, we aim to do experiments on large and more datasets with multiclass classification. We can also use different language datasets to perform text classification. It would be valuable to include emoticons as they are widely used in social media to represent expressions. Also, we will try to use the Twitter streaming API to retrieve tweets in real time in order to do a real-time sentiment analysis and explore other social networks.

## Figures and Tables

**Figure 1:** Research methodology.

**Figure 2:** Classification accuracy transfer learning-based approaches' results for fake news on COVID-19.

**Figure 3:** Classification accuracy transfer learning-based approaches results for COVID-19 English tweets.

**Figure 4:** Classification accuracy transfer learning-based approaches results for the extremist-non-extremist dataset.

**Figure 5:** Heat map of BERT-base.

**Figure 6:** Heat map of BERT-large.

**Figure 7:** Heat map of RoBERTa-base.

**Figure 8:** Heat map of RoBERTa-large.

**Figure 9:** Heat map of DistilBERT.

**Figure 10:** Heat map of ALBERT-base-v2.

**Figure 11:** Heat map of XLM-RoBERTa-base.

**Figure 12:** Heat map of Electra-small.

**Figure 13:** Heat map of BART-large.

**Figure 14:** Heat map of BERT-base.

**Figure 15:** Heat map of BERT-large.

**Figure 16:** Heat map of RoBERTa-base.

**Figure 17:** Heat map of RoBERTa-large.

**Figure 18:** Heat map of DistilBERT.

**Figure 19:** Heat map of ALBERT-base-v2.

**Figure 20:** Heat map of XLM-RoBERTa-base.

**Figure 21:** Heat map of Electra-small.

**Figure 22:** Heat map of BART-large.

**Figure 23:** Heat map of BERT-base.

**Figure 24:** Heat map of BERT-large.

**Figure 25:** Heat map of RoBERTa-base.

**Figure 26:** Heat map of RoBERTa-large.

**Figure 27:** Heat map of DistilBERT.

**Figure 28:** Heat map of ALBERTa-base-v2.

**Figure 29:** Heat map of XLM-RoBERTa.

**Figure 30:** Heat map of Electra-small.

**Figure 31:** Heat map of BART-large.

**Table 1:** Sample tweets of the COVID-19 fake news dataset.

Tweets	Labels
A chain lists recommendations to prevent and treat coronavirus	0
Australia closing borders in a few hours for 6 months	1

**Table 2:** Sample tweets of extremist-non-extremist dataset.

Tweets	Labels
Oh Allah, we are helpless	Nonextremist
Oh Allah, destroy US and Israel	Extremist

**Table 3:** Sample tweets of COVID-19 English tweets dataset.

Tweets	Labels
Bill Maher says coronavirus “overreactions” making him “sick:” “People die! That's what happens in life!	Uninformative
#Australia Melbourne GP clinic closed after doctor tests positive for #coronavirus after seeing 70 patients this month	Informative

**Table 4:** Transfer learning-based approaches results for fake news on COVID-19.

Model	Accuracy	Precision	Recall	*F*1 score
BERT-base	99.56	97.21	97.77	97.53
BERT-large	99.31	99.07	93.13	95.89
RoBERTa-base	99.71	99.85	96.84	98.29
RoBERTa-large	99.66	98.78	97.32	98.04
DistilBERT	99.41	96.69	96.69	96.69
ALBERT-base-v2	98.68	90.83	95.30	92.94
XLM-RoBERTa-base	99.22	96.01	95.08	95.54
Electra-small	99.17	96.85	93.56	95.14
BART-large	99.31	99.07	93.13	95.89

**Table 5:** Comparison of proposed approaches with state-of-the-art approaches.

State-of-the-art approaches				Proposed
[83]	[84]	[85]	[86]	Roberta-large
75%	93.6%	91%	91%	99.66%

**Table 6:** Transfer learning-based approaches results for COVID-19 English tweet dataset.

Model	Accuracy	Precision	Recall	*F*1 score
BERT-base	98.44	98.42	98.45	98.43
BERT-large	98.44	98.45	98.42	98.43
RoBERTa-base	96.48	96.48	96.62	96.48
RoBERTa-large	97.00	96.97	97.12	97.00
DistilBERT	98.31	98.39	98.23	98.30
ALBERT-base-v2	97.78	97.75	97.83	97.78
XLM-RoBERTa-base	98.57	98.53	98.61	98.56
Electra-small	94.52	94.66	94.76	94.52
BART-large	98.83	98.85	98.80	98.82

**Table 7:** Comparison of proposed approaches with state-of-the-art approaches.

State-of-the-art approaches		Proposed
[87]	[88]	Bart-large
0.78%	60.40%	98.83%

**Table 8:** Transfer learning-based approaches results for the extremist-non-extremist dataset.

Model	Accuracy	Precision	Recall	*F*1 score
BERT-base	99.71	98.82	97.84	98.33
BERT-large	99.71	98.82	97.84	98.33
RoBERTa-base	99.66	99.29	96.82	98.02
RoBERTa-large	99.36	98.56	94.16	96.24
DistilBERT	99.51	96.80	97.74	97.27
ALBERT-base-v2	98.97	94.80	93.45	94.12
XLM-RoBERTa-base	99.56	99.77	95.26	97.40
Electra-small	98.73	97.42	87.82	92.02
BART-large	99.56	98.22	96.77	97.48

**Table 9:** Comparison of proposed approaches with state-of-the-art approaches.

State-of-the-art approaches				Proposed
[89]	[90]	[91]	[92]	BERT-base/BERT-large
86.3%	85%	0.78%	76.5%	99.71%

## Data Availability

The data are not available until the thesis defense. In case of any queries, the readers can contact the corresponding author.
